The article "Comparison of TNFα to Lipopolysaccharide as an Inflammagen to Characterize the Idiosyncratic Hepatotoxicity Potential of Drugs: Trovafloxacin as an Example" was published in 2010. Journal: Int J Mol Sci.

# Comparison of TNFα to Lipopolysaccharide as an Inflammagen to Characterize the Idiosyncratic Hepatotoxicity Potential of Drugs: Trovafloxacin as an Example

**DOI:** 10.3390/ijms11114697

**Published:** 2010-11-18

**Authors:** Michael J. Liguori, Amy C. Ditewig, Jane F. Maddox, James P. Luyendyk, Lois D. Lehman-McKeeman, David M. Nelson, Vasanthi M. Bhaskaran, Jeffrey F. Waring, Patricia E. Ganey, Robert A. Roth, Eric A. G. Blomme

**Affiliations:** 1 Department of Cellular, Molecular, & Exploratory Toxicology, Abbott Laboratories; Abbott Park, IL 60064, USA; E-Mails: amy.ditewig@abbott.com (A.C.D.); jeff.waring@abbott.com (J.F.W.); eric.blomme@abbott.com (E.A.G.B.); 2 Department of Pharmacology & Toxicology, Center for Integrative Toxicology, Michigan State University; East Lansing, MI 48824, USA; E-Mails: maddox@cvm.msu.edu (J.F.M.); jluyendyk@kumc.edu (J.P.L.); ganey@cvm.msu.edu (P.E.G.); rothr@cvm.msu.edu (R.A.R.); 3 Discovery Toxicology, Bristol-Myers Squibb; Princeton, NJ 08540, USA; E-Mail: lois.lehman-mckeeman@bms.com (L.D.L.-M.); vasanthi.bhaskaran@bms.com (V.M.B.); 4 The Beatson Institute for Cancer Research, Glasgow, UK; E-Mail: d.nelson@beatson.gla.ac.uk

**Keywords:** idiosyncratic hepatotoxicity, liver, inflammation, rat, transcriptomics

## Abstract

Idiosyncratic drug reactions (IDRs) are poorly understood, unpredictable, and not detected in preclinical studies. Although the cause of these reactions is likely multi-factorial, one hypothesis is that an underlying inflammatory state lowers the tolerance to a xenobiotic. Previously used in an inflammation IDR model, bacterial lipopolysaccharide (LPS) is heterogeneous in nature, making development of standardized testing protocols difficult. Here, the use of rat tumor necrosis factor-α (TNFα) to replace LPS as an inflammatory stimulus was investigated. Sprague-Dawley rats were treated with separate preparations of LPS or TNFα, and hepatic transcriptomic effects were compared. TNFα showed enhanced consistency at the transcriptomic level compared to LPS. TNFα and LPS regulated similar biochemical pathways, although LPS was associated with more robust inflammatory signaling than TNFα. Rats were then codosed with TNFα and trovafloxacin (TVX), an IDR-associated drug, and evaluated by liver histopathology, clinical chemistry, and gene expression analysis. TNFα/TVX induced unique gene expression changes that clustered separately from TNFα/levofloxacin, a drug not associated with IDRs. TNFα/TVX cotreatment led to autoinduction of TNFα resulting in potentiation of underlying gene expression stress signals. Comparison of TNFα/TVX and LPS/TVX gene expression profiles revealed similarities in the regulation of biochemical pathways. In conclusion, TNFα could be used in lieu of LPS as an inflammatory stimulus in this model of IDRs.

## 1. Introduction

Idiosyncratic drug reactions (IDRs) represent a major threat to public health. These reactions are unpredictable, not readily detected in preclinical studies, and typically not uncovered until post-marketing of a drug after exposure of a large cohort of patients [1]. Typically, IDRs occur in a small subset of patients and are reversible upon removal of the drug. However, in many cases, the drug-induced severe liver damage results either in the need for a liver transplant or in fatality.

IDRs are likely the result of a complex interplay of genetic, environmental, and lifestyle factors [1]. Although unlikely to explain all IDRs, several hypotheses have been formulated for the mechanism(s) of these reactions. One such hypothesis postulates that a modest inflammatory episode can decrease the toxicity threshold of a drug, thus reducing its therapeutic index [2]. As such, drugs that are normally considered safe can cause significant adverse effects when associated with an inflammatory stimulus. This hypothesis was supported by the production of liver injury in rodent models in which bacterial lipopolysaccharide (LPS) was coadministered with drugs associated with hepatic IDRs, including diclofenac, ranitidine, chlorpromazine, sulindac, and trovafloxacin (TVX) [3–8].

The fluoroquinolone antibiotic, TVX, is a prototypical idiosyncratic hepatotoxicant with severe restrictions on its use [9]. Although TVX does not induce significant liver toxicity in rodents, it is toxic when coadministered with LPS as evidenced by increases in serum alanine aminotransferase activity (ALT) and hepatocellular necrosis [4,8]. Hepatic toxicogenomic analyses provide insight into toxic mechanisms [10], and these studies have shown that rats cotreated with TVX and LPS can be clearly differentiated from those treated with either agent alone, or cotreated with LPS and levofloxacin (LVX), a fluoroquinolone antibiotic not associated with liver toxicity in humans [4]. These observations were confirmed in an LPS mouse model [8,11,12].

Although the rodent LPS/TVX models represent valuable research tools for in-depth mechanistic studies, their major shortcomings are related to the variability associated with the heterogeneous nature of LPS. The central domain of LPS consists of a glycolipid (lipid A) and a polysaccharide moiety, which can further be subclassified into a core oligosaccharide and an O-specific polysaccharide (OPS) [13]. This OPS substituent can have long polysaccharide repeats with a variety of possible monosaccharide components, resulting in significant structural and biological diversity among bacterial species and preparations of LPS. As a consequence, the use of LPS as a principal inflammagen requires time-consuming, dose range finding studies and makes it difficult to develop a standardized protocol.

In an attempt to establish a standardized protocol for this model of IDRs, we evaluated a surrogate modulator of inflammation, tumor necrosis factor-α (TNFα), to replace LPS. TNFα is a member of a superfamily of inflammatory mediators involved with immunogenic responses to a variety of pathogens [14]. The cellular functions of TNFα are diverse and include activation of apoptosis via “death receptors”, initiation of an inflammatory signal partially by influencing the conformation of adhesion molecules, cell proliferation and differentiation, and protection from infection [15]. Its endogenous regulation is complex and involves a myriad of cell types, predominantly macrophages, Kupffer cells, T-cells, and neutrophils for its production and effects. This cytokine can be produced as a recombinant protein with homogenous composition.

In the LPS/drug models studied thus far, TNFα activation appears to be a critical, proximal event in initiating a cascade of downstream inflammatory events that ultimately result in hepatocellular necrosis [16,17]. Indeed, cotreatment of mice with TNFα and TVX resulted in liver injury similar to that seen after coadministration of LPS and TVX [17]. Replacement of LPS with TNFα might avoid variability due to the marked differences in biological activity associated with LPS preparations. Accordingly, the present study focused on the evaluation of rat recombinant TNFα compared to LPS, both alone and in combination with TVX. Specifically, the objectives were (1) to compare, in rats, the hepatic transcriptomes induced by treatment with LPS or TNFα, (2) to evaluate toxicity induced by combination dosing using TNFα/TVX or TNFα/LVX, and (3) to compare the effects induced by TNFα/TVX versus LPS/TVX.

## 2. Results and Discussion

### 2.1. Results

#### 2.1.1. Serum Chemistry and Histopathology for the TNFα Study

TNFα treatment (0.01 mg/kg i.v.) resulted in no evidence of acute liver injury after 6 hours exposure in three separate studies (3 rats per study; total n = 9 rats) using 3 different lots of TNFα. No significant changes in liver enzyme activities (ALT, AST, GGT, ALP) were evident. No histologic changes were identified in the liver.

#### 2.1.2. Comparison of Hepatic Transcriptomes Induced by LPS or TNFα

TNFα treatment resulted in extensive (∼2700) global liver transcriptomic changes. These changes were consistent among individual studies, lot numbers, and animals (Figure 1A, B) as evidenced by hierarchical cluster analysis and principal component analysis (PCA) of individual global expression profiles. The heatmap in Figure 1A shows that the profiles from two separate preparations of TNFα were indistinguishable from a third preparation. Using PCA, the liver profiles from all TNFα-treated rats were localized into one cluster, suggesting a high degree of similarity between the three lots with low inter-individual variability (Figure 1B). A complete listing of gene expression changes is presented in supplemental Table 1.

LPS treatment also induced a large number of gene expression changes (∼5600). Unlike TNFα, the LPS lots induced different transcriptomic responses (Figure 1A, B). In particular, PCA clustering separated the expression profiles based on the lot of LPS used in each study. Individual animals dosed with the same lot of LPS displayed little variability, indicating that the major component of variation was due to LPS lot differences rather than inter-individual variation. It should be noted that these studies were conducted independently, which may also contribute to variability. Although these gene expression variations were evident, LPS did not result in significant liver injury (as measured by serum chemistry and histopathology) in either study at the early time evaluated (t = 4 h). The clusters resulting from the expression profiles of LPS-treated rats (Figure 1B) were distinct from those treated with TNFα, and the overall number of expression changes was much greater than those induced by TNFα. The Venn diagram in Figure 2 illustrates the large number of LPS-induced expression changes. Of these, 16% overlapped with TNFα-induced changes, but the majority of the LPS changes were distinct. In contrast, 54% of the TNFα-induced transcriptional changes overlapped with those induced by LPS.

#### 2.1.3. Classification of Biochemical Pathways Significantly Impacted by LPS or TNFα

Classification of genes into their corresponding biochemical pathways can give insight into underlying biological function. Individual hepatic gene expression profiles from LPS or TNFα-treated rats were combined in silico to reduce inter-individual variability and to increase stringency, and these genes were classified and ranked into the corresponding pathways. The analysis separated the pathways into those perturbed by both LPS and TNFα (Figure 3A, B) and by those changed solely by each respective agent (Figure 3C, D). For those impacted by both LPS and TNFα (*i.e.*, mostly driven by the 731 overlapping genes shown in Figure 2), most of the pathways were involved with various immunological processes. However, there were differences in the magnitude of perturbation by each treatment. For LPS, ER-stress response and interferon signaling ranked highest (∼40–50%) followed by multiple immune and cytokine pathways with impact values >20% (most genes were upregulated). For TNFα, similar immune pathways were impacted, but they differed in rank ordering with lower percent impact and included more downregulated genes (Figure 3B, D). Besides immune and inflammatory responses, LPS and TNFα perturbed pathways involved with various stress response signals, including those involved with stellate cell activation and hepatic cholestasis.

Whereas expression changes after treatment with LPS or TNFα exhibited many similarities, the overall pathway impact resulting from LPS treatment was more robust and extensive (increased percent perturbation), consistent with the Venn analysis. Several pathways perturbed uniquely by LPS were involved with apoptotic and death receptor signaling. These results suggest that LPS has a greater effect overall compared to TNFα on inflammation signals in liver at the doses and the timepoint evaluated.

#### 2.1.4. Evaluation of Fluoroquinolone Toxicity after TNFα Coadministration

Rats given TNFα alone, TVX alone, LVX alone, or any combination of TNFα and fluoroquinolone showed no significant changes in serum chemistry, and there were no significant liver histopathology findings (data not shown).

TVX or LVX alone induced few (∼300–500) gene expression changes (|fold change| ≥ 2; p ≤ 0.01), suggesting a minor impact on overall liver homeostasis (Figure 4A). Treatment with TNFα/LVX or TNFα/TVX resulted in a pronounced increase in hepatic gene expression changes (∼2500 and 3500 respectively for each co-dose) relative to treatment with TNFα or either agent alone. Cluster analysis indicated that the TNFα/TVX-induced expression profiles were significantly different from those of all other treatment groups. For the livers from TNFα/TVX-treated rats, rigid selection criteria distinguished 679 probe sets that were uniquely regulated (Figure 4B). This subset of genes included the neutrophil (PMN) chemokines, CINC-1 (∼40-fold increase) and MIP-2 (∼7-fold increase) (Figure 5A), which were previously reported to be increased in the LPS/TVX model of hepatotoxicity [4]. In contrast, TNFα alone and TNFα/LVX treatments regulated <∼100 probe sets.

Interestingly, TNFα/TVX treatment resulted in a marked autoinduction of TNFα expression, which was not observed in any other treatment group (Figure 5B). TNFα overstimulation was also reflected in an extensive induction of downstream signaling members of the TNFα cascade (Figure 6). In contrast, this pathway was not affected in livers from TNFα/LVX treatment (data not shown).

#### 2.1.5. Comparison of Gene Expression Profiles Induced by TNFα/TVX and LPS/TVX

Gene expression profiles from the livers of TNFα/TVX-treated rats formed a unique cluster relative to rats treated with TNFα alone and to TNFα/LVX-treated rats, a result similar to the pattern observed with LPS/TVX treatment. Upregulation of PMN chemokines (CINC-1 and MIP2) was similar between the TNFα and LPS models, but LPS/TVX did not induce TNFα over LPS alone (Figure 5B).

In Tables 1–3, a rank ordering (as determined by Ingenuity Pathways software) was completed for the top (p < 0.06) biochemical pathways impacted by the unique gene expression changes induced by TNFα/TVX and/or LPS/TVX cotreatment, but not by each drug, TNFα, or LPS alone. Of these, 11 pathways were impacted similarly by TNFα/TVX and LPS/TVX cotreatments (Table 1), including tight junction networks, fMLP signaling in PMNs, IL-12 signaling, and p53 signals. Some notable pathways impacted only by TNFα/TVX (Table 2) included ATM signaling, hypoxia signaling, cell cycle control, NF-κB signaling, cytokine signaling, and response to ROS. Finally, unique pathways changed only in livers from LPS/TVX-cotreated rats (Table 3) included MAPK signals, cytokine communication, mitochondrial dysfunction, PDGF signaling, toll-like receptor, and mRNA processing. Although there were several specific pathway differences between the two treatment groups, the overall function/theme of many pathways overlapped, which suggested a similar innate immune system-enhancing effect from the presence of TVX after pretreatment with either LPS or TNFα.

### 2.2. Discussion

One proposed mechanism to explain some IDRs is that a mild underlying inflammatory stimulus lowers the therapeutic index for an otherwise safe drug [2]. Although this mechanism is unlikely to explain all IDRs, background information on a compound’s potential to exacerbate inflammation may be useful toward risk assessment of compounds in preclinical development. Currently, the most characterized inflammatory agent used to address the proposed mechanism is LPS [2,4,16]. LPS is a potent activator of the immune system and leads to a massive stimulation of gene transcription, especially in the bone marrow, spleen, and liver [18].

LPS is a useful inflammagen for mechanistic evaluation of drugs with known liabilities. However, the heterogeneous nature of LPS renders difficult the establishment of a standardized test protocol. Gene expression profiling confirmed that different preparations of LPS caused significantly different hepatic transcriptomic responses that were not attributable to individual animal variation. In contrast, TNFα resulted in remarkably consistent transcriptomic profiles regardless of preparation. Therefore, replacing LPS with TNFα could provide a model with enhanced reproducibility, reducing the need for extensive dose range finding studies.

In previous model characterizations, acute exposure to LPS at the doses used resulted in no overt liver injury [4]. Likewise, acute dosing with TNFα yielded no significant changes in serum chemistry or histology under these experimental conditions despite a clear signal at the level of transcription. The lack of a phenotypic effect is likely due to the acute dosing period (<6 h) and to the small dose administered. Both proinflammatory agents induced similar changes in several cell signaling networks, especially those related to innate immune response pathways. However, the LPS effects were broader, as evidenced by the greater number of pathways impacted and a more pronounced level of gene regulation.

LPS and other bacterial products mediate their effects partly via stimulation of toll-like receptors (TLRs), resulting in signal transduction and synthesis of various immune activators, such TRAF and NF-κB [19]. This results in rapid mobilization of immune mediators to the primary infection sites. LPS itself, via activation of receptors such as TLR4, mediates signaling to downstream MAP3Ks, which in turn are essential for secretion of native TNFα and for the subsequent innate immune response [20,21]. TNFα biosynthesis results from LPS stimulation of cells, and this cytokine mediates some of the effects produced by LPS. However, LPS stimulates activation of additional immune mediators, including IL-6 [22], IL-12 [23], MCP-1 [24], and IL-8 [25]. Therefore, the enhanced perturbation of gene expression by LPS relative to TNFα is not surprising.

Globally, TNFα/TVX treatment resulted in greater changes in the liver transcriptome compared to TNFα/LVX, despite the fact that LVX was administered at a 5-fold greater dose (comparable to the fold-difference in doses used clinically). From the TNFα/TVX group, genes involved with NF-κB activation such as RELA and TRAF2 were significantly induced. NF-κB activation occurs as a response to inflammatory stimuli and is integrally linked to TNFα signaling [26] TRAF2 regulates these signals via ubiquitin ligation to its targets (IκB), which releases NF-κB to exert its effects [27]. All of these perturbations were absent in the TNFα/LVX unique gene set, suggesting that the ability of TVX to potentiate an innate immune response is not shared by LVX. This supports the feasibility of evaluating novel drug development candidates for their ability to enhance an underlying inflammatory stimulus. Evaluation of additional IDR-inducing molecules would aid in the validation of such a model.

TNFα, acting through its receptors (TNFR1 and TNFR2), is a critical mediator for manifestation of TVX hepatotoxicity in LPS-treated mice [8,28]. Indeed, cotreatment with TNFα and TVX produced liver injury in mice [17]. Gene array data might facilitate elucidation of key mechanism(s) in this interaction. Furthermore, data from mice further support the choice of TNFα itself as an appropriate external inflammatory stimulus for these rodent models.

Also critical to the evaluation of the use of TNFα in lieu of LPS were the comparisons between TNFα/TVX and LPS/TVX responses. Unlike the mouse, there was no evidence of overt liver toxicity following TNFα/TVX administration at the early timepoint evaluated. The lack of a phenotypic effect at this early timepoint may reflect on the inability of TNFα to activate inflammatory signal transduction to the same extent as LPS in rats. The lack of an overt signal in rat may also suggest that mice are a more sensitive species to a TNFα/TVX interaction. For interpretation of gene expression data, early timepoints offer the advantage of enhanced insight into potential primary mechanisms of action. Indeed, genome-wide mRNA profiling of livers from TNFα/TVX-treated rats suggested a remarkable similarity in mode of action when compared to LPS/TVX in rats. More specifically, TNFα/TVX and LPS/TVX treatment perturbed similar immunological and stress response pathways, thus suggesting, despite differences in signaling robustness with no visible early injury, that treatment with LPS or TNFα ultimately led to similar toxicogenomic outcomes. Robust gene expression signals, such as those observed with TNFα/TVX treatment, are considered predictive of subsequent injury [10]. In addition, although a number of specific pathways did overlap between TNFα/TVX and LPS/TVX, a more important factor may be that TNFα/TVX cotreatment activates the necessary/key pathways that may contribute to liver pathogenesis.

Coadministration of TNFα/TVX resulted in marked autoinduction of TNFα mRNA, which was absent upon exposure to TNFα alone or TNFα/LVX. Transactivation of factors downstream of the TNFα receptor substantiated this observation for the TNFα/TVX-cotreated rats. Autoinduction could potentially perpetuate inflammatory cascades and immune cell activation. Indeed, in the mouse model, there is evidence for dysregulated amplification cycles in which TNFα enhances expression of other inflammatory cytokines, leading to further TNFα production [17]. This could eventually augment the presence of deleterious factors resulting in toxicity. In mice, TVX has been shown to be a critical mediator of hepatotoxicity at least partially through sustained TNFα signaling [17]. TNFα/TVX cotreatment primarily reduced the clearance of endogenous serum TNFα with a relatively smaller effect of increased production. This was a rare example of a xenobiotic reducing systemic clearance of a cytokine. In that mouse study, mRNA expression of hepatic TNFα was not evaluated. Here, using gene expression analysis, we showed that enhanced expression in liver represents one source of increased TNFα in serum. Interestingly, hepatic gene expression of TNFα was not elevated in livers of LPS/TVX–treated animals compared to those treated with LPS alone, suggesting that other factors also contribute to the toxicity. However, we cannot exclude the possibility that the failure to observe an influence of TVX on TNFα expression in LPS-cotreated rats was due to pharmacokinetic differences, *i.e.*, differences in the time of initial TNFα exposure relative to sacrifice time in the LPS- and TNFα-cotreated groups.

The exact mechanism responsible for the TVX-induced autoinduction of TNFα is unknown and requires further investigation. Understanding this mechanism could lead to further insight into understanding TVX-induced hepatotoxicity since inflammatory mediators have been clearly linked to certain hepatotoxicities [29]. Relatively few reports exist describing this autoinduction effect. TNFα increases its own expression in some in vitro systems like human ZR-75-1 breast cancer cells [30] and rat tracheal epithelial cells [31]. In HL60 leukemia cells, autoinduction of TNFα required phospholipase A_2_ and lipoxygenase activity with subsequent release of arachidonic acid metabolites [32]. In the present study, phospholipase A_2_ activating protein (Plaa) mRNA was overexpressed in the TNFα and TNFα/TVX treated rats, but was not consistently increased in the TNFα/LVX group. No change was observed in lipoxygenase expression, but phospholipase A_1_ (Pla1a) was increased in all rats treated with TNFα either alone or in combination with TVX or LVX.

## 3. Experimental Section

### 3.1. Administration of TNFα and Fluoroquinolone Drug

All animal experiments for this study were conducted in accordance with the Guiding Principles in the Use of Animals in Toxicology (Anonymous 2002) and were approved by Abbott’s Institutional Animal Care and Use Committee (IACUC). Male Sprague-Dawley rats [Crl:CD^®^(SD)IGS BR], weighing ∼250 g at study initiation were obtained from Charles River Laboratories, Inc. (Wilmington, MA). Rats were housed singly in ventilated, stainless steel, wire-bottom hanging cages and fed non-certified Rodent Chow (Harlan Labs, Madison, WI) and water ad libitum.

After 24 h fasting, the rats were injected with recombinant rat TNFα (Sigma Chemical, St Louis, MO; lot numbers 126K1053, 087K1290, or 098K1865) via tail vein (i.v.) at a dose of 0.01 mg/kg body weight with a delivery volume of 1 mL/kg. This dose of TNFα was based on rat studies contained in the DrugMatrix™ database [33]. For the lot comparison analysis, TNFα was given in separate studies which were conducted several months apart. Two hours after TNFα administration, rats were treated (i.v.) with TVX (30 mg/kg), LVX (150 mg/kg) or vehicle (dextrose 5% in water with 0.1 N equivalent HCl) in a volume of 5 mL/kg. The previous LPS rat model served as a basis for dose selection with a lower TVX dose due to formulation restriction [4]. Treatment nomenclature was designated as follows: Veh/Veh (n = 3), TNFα/Veh (n = 9), Veh/TVX (n = 3), Veh/LVX (n = 3), TNFα/TVX (n = 3), and TNFα/LVX (n = 3). TNFα (lot #126k1053) was used for coadministration with TVX and LVX. Four hours after the second treatment, the rats were sacrificed using CO_2_ anesthesia and blood was collected. A portion of the liver was flash frozen in liquid nitrogen, and the remaining liver was preserved in 10% neutral-buffered formalin. One TNFα/LVX rat was misdosed and was therefore excluded from further analysis.

### 3.2. Administration of LPS

Two different lots of LPS were used to compare hepatic gene expression changes. These studies were conducted at Michigan State University (MSU, East Lansing, MI) using a protocol similar to that previously described [4]. Rats received humane care according to the criteria outlined in the Guide for the Care and Use of Laboratory Animals (1996) prepared by the National Academy of Sciences, and procedures were approved by the Michigan State University Committee on Animal Use and Care. Male Sprague-Dawley rats [Crl:CD (SD)IGS BR; Charles River, Portage, MI] (n = 5) weighing 250–350 g were used for these studies. Animals were fed standard chow (rodent chow/Tek 8640; Harlan Teklad, Madison, WI) and allowed access to water ad libitum. In one study, LPS derived from Escherichia coli serotype O55:B5 with an activity of 9.2 × 10^6^ EU/mg was used (catalog number L-2880, Lot 024K4067; Sigma-Aldrich, Inc., St. Louis, MO), designated in Figure 1 as Lot #2. This activity was determined using a QCL Chromogenic LAL Endpoint Assay from Cambrex (East Rutherford, NJ). Rats fasted for 24 h were given 44.4 × 10^6^ EU/kg LPS or its saline vehicle (Veh) i.v., and food was then returned. Two hours later, vehicle (50/50 sterile saline/sterile water) was administered i.v. Two hours later, rats were anesthetized with sodium pentobarbital (75 mg/kg i.p.) and euthanized by exsanguination. The right medial lobe of the liver was flash-frozen in liquid nitrogen for subsequent gene expression analysis. For Lot #1 in Figure 1 (Lot 51K4115), data files were used from a previously published study [34] in which rats were treated with LPS (from *E. Coli*, serotype 055:B5) and vehicle using the same dose (44.4 × 10^6^ EU/kg LPS) and treatment protocol as described for Lot #2.

### 3.3. Serum Chemistry and Histopathology for the TNFα Study

Serum clinical chemistry parameters for the TNFα study were quantified using an Aeroset Clinical Chemistry Analyzer (Abbott Laboratories, Abbott Park, IL) and included: alanine amino transferase (ALT), aspartate amino transferase (AST), gamma glutamyltransferase (GGT), and alkaline phosphatase (ALP) activities. Formalin-fixed liver samples (left and right lobes) were embedded in paraffin and sections (6 μm) were stained with hematoxylin and eosin.

### 3.4. RNA Preparation

Frozen liver samples (approximately 100 mg of tissue per sample) were immediately added to 2 mL of QIAzol reagent (Qiagen, Valencia, CA) and homogenized using a Polytron 300D homogenizer (Brinkman Instruments, Westbury, NY). One mL of the tissue homogenate was transferred to a microfuge tube, and total RNA was extracted via chloroform extraction followed by nucleic acid precipitation with isopropanol. The pellet was washed with 80% ethanol and resuspended in molecular biology grade water. Nucleic acid concentration was determined by O.D. 260 nm (Smart-Spec; Bio-Rad Laboratories, Hercules, CA), and RNA integrity was evaluated using a bioanalyzer (model 2100; Agilent Technologies, Foster City, CA).

### 3.5. Gene Array Analysis

Microarray analysis of rat liver samples was performed using the standard protocol provided by Affymetrix, Inc. (Santa Clara, CA) as previously described [4] using Affymetrix Rat Genome RAE 230_2.0 or RAE230A arrays containing ∼31,000 or ∼15,000 probe sets (genes) respectively. Resolver software (Version 7.2; Rosetta Informatics, Seattle WA) was used to analyze the microarray data (available in supplemental Table 1). Ingenuity Pathways Analysis software (Version 8.0 Ingenuity Systems, Redwood City, CA) was applied for pathway evaluations. For TNFα/TVX comparisons to LPS/TVX, the original data files from the previous LPS/TVX study were used [4].

### 3.6. Statistics and Pathway Analysis

Clinical pathology parameters and mRNA fold changes were analyzed by analysis of variance (ANOVA) with Tukey’s post hoc test using GraphPad Prism software (Version 5; La Jolla, CA). The criterion for significance was p ≤ 0.05. For hepatic microarray analysis, the scanned image and intensity files (.cel files) were imported into Resolver software. Gene expression ratios were built for each drug-treated animal versus the respective vehicle-treated animals combined in silico using the Resolver error model. All hierarchical cluster and principal component analyses were completed with Resolver software. Gene expression data for each rat were entered into Ingenuity software (combined in silico), which then ranked and calculated percent pathway impact (number of genes regulated/total number of genes in pathway) with a corresponding p-value for each treatment. Pathways impacted similarly and differentially upon exposure to the respective treatment were identified. In a given analysis, the number of genes/probe sets represented depends on the statistical cutoffs and stringency parameters for each separate analysis, resulting in a slightly different magnitude of probe sets presented. All analysis cutoffs are listed in each figure description.

## 4. Conclusions

The results here describe a new rat model of IDR using TNFα that could support preclinical characterization of certain new drug candidates. Transcriptomic characterization of the model revealed a consistent hepatic response upon TNFα pretreatment. Further characterization of the model with the IDR-inducing drug TVX resulted in a sustained autoinduction of TNFα. This enhanced inflammatory response could be a component in the hepatotoxicity induced by TVX.

## Supplementary Data



## Figures and Tables

**Figure 1.** (**A**) Comparison of the hepatic gene expression profiles for LPS- or TNFα-treated rats using separate lots of each agent. Individual probe sets (genes) are displayed on the horizontal axis and each individual treatment is on the vertical axis. Shades of red indicate increased expression relative to the vehicle (Veh) treatment, and shades of green indicate decreased expression. Black indicates no statistically significant change in expression. Both the genes and experiments were analyzed using divisive hierarchical cluster analysis with Euclidean distance as the similarity measure. The dendogram shows relative similarities between the individual expression profiles. Statistical filters were applied using |fold change| ≥ 2.0 and p ≤ 0.01 in at least one rat. Number of probe sets represented in each heatmap is TNFα (∼2700) and LPS (∼5600). Lot designations: TNF Lot #1 (098K1865); TNF Lot #2 (126K1053); TNF Lot #3 (087K1290); LPS Lot #1 (51K4115); LPS Lot #2 (024K4067). (**B**) Principal component analysis (PCA) of liver gene expression profiles for all TNFα-treated and LPS-treated rats. Three principal components were generated and plotted for each expression profile (|fold change| ≥ 2.0 and p ≤ 0.01) using Rosetta Resolver software. Treatments that clustered together are represented within the same oval.

**Figure 2.** Venn diagram comparing the liver gene expression changes induced by TNFα or LPS treatment (|fold change| ≥ 2.0 and p ≤ 0.05). Individual gene expression changes were combined in silico for this comparison.

**Figure 3.** Results of Ingenuity Pathway Analysis for rats treated with either LPS or TNFα. Ingenuity software was applied to classify the top pathways that were impacted after treatment. To account for inter-individual variability, gene expression profiles from each TNFα- or LPS-treated rat were combined in silico using Resolver software. From these combined groups, genes with |fold change| ≥ 2.0 and p ≤ 0.05 were evaluated in the pathway analysis. Pathways were separated into those perturbed by both LPS and TNFα (Panel A/B) and by those changed uniquely by each respective agent (Panel C/D). Pathway names are listed on the y-axis and percent impact is listed on the x-axis. Each bar is subdivided to indicate the relative percentage of upregulated (red) vs. downregulated (green) genes. P-values were also generated as indicated by the black line using the entire array as the background set. (**A**) Pathway analysis of the genes differentially expressed in the liver upon treatment of rats with LPS: these pathways were also changed by treatment with TNFα. The 731 overlapped genes (Figure 2) are the major component of these pathway changes. (**B**) Pathway analysis of the genes differentially expressed in the liver upon treatment of rats with TNFα: these pathways were also changed by treatment with LPS (panel A). Since these pathways were also impacted by LPS, they are listed in the same order as panel A for ease of comparison. (**C**) LPS-specific pathways were identified for the genes differentially expressed in the liver. These pathways were not perturbed by TNFα. The 3949 LPS-specific genes (Figure 2) are the major component of these pathway changes. (**D**). TNFα-specific pathways were also identified for the genes differentially expressed in the liver. These pathways were not perturbed by LPS. The 631 TNFα-specific genes (Figure 2) are the major component of these pathway changes.

**Figure 4.** (**A**) Hierarchical cluster analysis of hepatic gene expression profiles induced by cotreatment with the following agents: Veh/TVX, Veh/LVX, TNFα/Veh, TNFα/LVX, or TNFα/TVX. TNFα/drug cotreatment was completed with only one TNFα lot (see Experimental Section). The dendrogram indicates that the TNFα/TVX treatment is unique compared to all other groups. Statistical filters were applied using |fold change| ≥ 2.0 and p ≤ 0.01. (**B**) A Venn diagram overlapping the gene expression profiles induced in the liver of rats by TNFα/TVX, TNFα/LVX, and TNFα/Veh. Stringent gene filtration criteria (|FC| ≥ 1.5 & p ≤ 0.05 in 2 of 3 rats) were used to remove genes with high biological variation. The TNFα/TVX treatment uniquely regulated the largest number of genes (679).

**Figure 5.** (**A**) Comparison of the relative mRNA expression for the neutrophil chemokines (MIP2 and CINC1). Each bar represents treatment with Veh, TVX, or LVX and cotreatment with either Veh or TNFα. The y-axis represents fold change of mRNA level vs. vehicle. The expression profiles from each individual rat were pooled in silico using Rosetta Resolver software (gene expression change p < 0.05) to account for inter-animal variation. Error bars represent standard deviation. * Significantly different from Veh/Veh and TNFα/Veh (p < 0.05); # Significantly different from Veh/Veh; ** Significantly different from Veh/Veh, but not from TNFα/Veh; ## Significantly different from Veh/Veh and TNFα/Veh. (**B**) Quantitation of endogenous hepatic TNFα mRNA with or without exposure to exogenous TNFα protein. Labels and inter-animal variation are the same as in panel A. TNFα/TVX treatment shows a large autoinduction of TNFα mRNA. * Significantly different from Veh/Veh, TNFα/Veh, TNFα/LVX (p < 0.05); ** Significantly different from Veh/Veh.

**Figure 6.** Effect of TNFα autoinduction on the expression of members downstream from TNFα signal transduction. Pathway diagram was generated using Ingenuity software. Each pathway member labeled in red or green represents upregulation or downregulation, respectively. White represents no significant change in expression. TNFα/TVX showed a large degree of downstream activation in contrast to TNFα/LVX (data not shown).

**Table 1.** List of Biochemical Pathways Regulated in Common Between TNFα/TVX and LPS/TVX.

**Both TNFα/TVX & LPS/TVX**				
**Pathway Name**	**TNF/TVX % Impact**	**TNF/TVX P-Value**	**LPS/TVX % Impact**	**LPS/TVX P-Value**
Tight Junction Signaling	26.1%	0.001	18.5%	0.021
MIF Regulation of Innate Immunity	33.3%	0.003	22.2%	0.039
Dendritic Cell Maturation	25.3%	0.004	20.0%	0.013
NFAT Regulation of Immune Response	24.4%	0.011	17.9%	0.058
fMLP Signaling in Neutrophils	26.2%	0.013	19.7%	0.051
IL-12 Signaling in Macrophages	23.9%	0.018	20.9%	0.014
Glucocorticoid Receptor Signaling	20.5%	0.021	17.9%	0.012
p53 Signaling	22.0%	0.025	22.0%	0.004
B Cell Receptor Signaling	20.5%	0.040	18.2%	0.023
Role of Macrophages, Fibroblasts and Endothelial Cells in RA	18.3%	0.040	17.6%	0.005
Molecular Mechanisms of Cancer	17.8%	0.044	14.9%	0.043

**Table 2.** List of Biochemical Pathways Regulated by TNFα/TVX, but not by LPS/TVX.

**TNFα/TVX**		
**Pathway Name**	**% Impact**	**P-Value**
ATM Signaling	34.4%	0.001
Hypoxia Signaling in the Cardiovascular System	32.0%	0.001
Cell Cycle: G2/M DNA Damage Checkpoint Regulation	37.0%	0.002
CD28 Signaling in T Helper Cells	27.9%	0.003
HMGB1 Signaling	27.0%	0.004
Role of PKR in Interferon Induction and Antiviral Response	32.3%	0.006
Androgen Signaling	26.1%	0.007
Activation of IRF by Pattern Recognition Receptors	27.8%	0.008
NF-κB Signaling	23.8%	0.009
IL-10 Signaling	27.5%	0.010
CD27 Signaling in Lymphocytes	27.3%	0.010
p38 MAPK Signaling	24.2%	0.012
4-1BB Signaling in T Lymphocytes	31.8%	0.013
Death Receptor Signaling	25.0%	0.017
Cholecystokinin/Gastrin-mediated Signaling	24.2%	0.024
iCOS-iCOSL Signaling in T Helper Cells	24.5%	0.025
Relaxin Signaling	23.5%	0.025
Role of BRCA1 in DNA Damage Response	25.0%	0.026
Role of RIG1-like Receptors in Antiviral Innate Immunity	27.3%	0.026
Production of Nitric Oxide and ROS in Macrophages	21.5%	0.028
ILK Signaling	21.1%	0.031
Cdc42 Signaling	21.4%	0.040
Angiopoietin Signaling	25.0%	0.042
AMPK Signaling	23.8%	0.045
Pattern Recognition Receptors in Bacteria/Virus	20.5%	0.046
Phospholipase C Signaling	17.9%	0.049
Hepatic Cholestasis	19.8%	0.050
Protein Kinase A Signaling	18.5%	0.060
B Cell Activating Factor Signaling	24.0%	0.062

**Table 3.** List of Biochemical Pathways Regulated by LPS/TVX, but not by TNFα/TVX.

**LPS/TVX**		
**Pathway Name**	**% Impact**	**P-Value**
Chronic Myeloid Leukemia Signaling	23.1%	0.006
LPS-stimulated MAPK Signaling	25.5%	0.006
PDGF Signaling	23.4%	0.017
Communication between Innate and Adaptive Immune Cells	25.0%	0.018
PPAR Signaling	21.9%	0.019
VDR/RXR Activation	23.1%	0.026
Cytokines in Mediating Communication between Immune Cells	31.2%	0.028
Toll-like Receptor Signaling	20.0%	0.031
GM-CSF Signaling	24.4%	0.032
Cleavage and Polyadenylation of Pre-mRNA	37.5%	0.034
Fc Epsilon RI Signaling	19.6%	0.039
Cell Cycle: G1/S Checkpoint Regulation	20.5%	0.044
Estrogen Receptor Signaling	18.2%	0.046
T Cell Receptor Signaling	18.9%	0.049
CD40 Signaling	21.1%	0.051
Wnt/β-catenin Signaling	17.4%	0.051
PI3K/AKT Signaling	18.3%	0.056
TREM1 Signaling	21.9%	0.056
Regulation of eIF4 and p70S6K Signaling	19.1%	0.058
Mitochondrial Dysfunction	17.6%	0.062
Cell Cycle Regulation by BTG Family Proteins	25.0%	0.063

## Non-Standard Abbreviations:

IDR: Idiosyncratic drug reaction
LPS: lipopolysaccharide
TNFα: tumor necrosis factor-α
TVX: trovafloxacin
LVX: levofloxacin
OPS: O-specific polysaccharide
ALT: alanine amino transferase
AST: aspartate amino transferase
GGT: gamma glutamyltransferase
ALP: alkaline phosphatase
TBIL: total bilirubin
PCA: principal component analysis
interferon: IFN
PMN: neutrophil
ER: endoplasmic reticulum
ROS: reactive oxygen species
MAP3Ks: mitogen-activated protein kinase kinase kinase
IL-12: interleukin-12
ATM: ataxia telangiectasia-mutated
